# Cross-Media Narrative and Emotional Identity Mechanism of School Culture in Media Integration Environment

**DOI:** 10.1155/2022/5017227

**Published:** 2022-09-10

**Authors:** Anmin Jia

**Affiliations:** School of Chinese Languages and Literature, Shanxi University, Taiyuan 030006, China

## Abstract

Cross-media narrative of school culture is essentially different from emotional identity. We cannot just rely on students' rote learning to achieve this teaching goal, but we must let students gradually deepen their learning experience in the learning process. As a new narrative form in the context of media convergence, its narrative strategy from the perspective of media convergence culture can promote the industrialization of IP cultural resources, such as content production, marketing and dissemination, and derivatives development. This paper mainly studies the cross-media narrative and emotional identity of school education culture through wavelet transform algorithm. The research shows that the error rate of this paper is the lowest among the three methods, with the highest error rate of 46.8%, followed by the method of literature Sara 2018 with the highest error rate of 64.8%, and finally the method of literature Neate et al. 2017 with the highest error rate of 71.8%. It can be seen that this method is the most suitable for identifying the emotional characteristics of school education culture. Through wavelet transform, teachers can infiltrate the basic knowledge of Chinese into the cultivation of students' emotions in the teaching process, which is conducive to students' emotional edification, personality development, and self-motivation.

## 1. Introduction

The significance of school education culture lies in swearing in the ideology of education practice, in seeking individualized education understanding, and in the mode of thinking and behavior of school education practice, in order to clarify the spiritual pursuit of the school and form a common vision leading to the sustainable development of the school. As a new form of narration in the context of media integration, the emergence of the concept of cross-media narration and its related discussions are receiving more and more attention, and its cultural and market development value is also increasingly apparent. Its narrative strategy from the perspective of media integration culture plays a sustainable role in promoting the industrialization of IP cultural resources, such as content production, marketing and dissemination, and derivatives development [1]. The cross-media narration of school education culture is fundamentally different from emotional identity. Students cannot only rely on rote learning to achieve this teaching goal. Students must gradually deepen their learning experiences in the learning process, so as to arouse the resonance of students in emotional education, promote the progress and development of junior middle school Chinese teaching, and improve students' comprehensive quality for their future learning to lay a solid foundation for life. Cross-media narration and emotional education meet the fundamental requirements of quality education and embody the connotation of quality education [2, 3]. It integrates psychology and pedagogy and applies them to Chinese teaching in junior middle school, for better connecting of teachers' emotions with students' emotions, which can effectively strengthen the relationship between teachers and students. The emotional education of school education culture is an educational concept that conforms to the characteristics of the times. It perfectly integrates pedagogy and psychology and acts on the teaching of students [4]. Adopting emotional education can not only promote students' learning interest and initiative but also further enhance the teacher-student relationship in emotional teaching activities and promote teachers' further understanding of students, which will also be of great help to the next teaching activities.

There are three main viewpoints of school education culture: one is the theory of natural growth, the other is the theory of inheritance and innovation, and the third is the theory of active construction. The unreliability of the “natural growth theory” lies in the reason that why school culture can communicate is due to “speech”, and the subjectivity of “speech” is contrary to natural growth. Therefore, this paper mainly studies the cross-media narrative and emotional identity of school education and culture through the wavelet transform algorithm. The main principle of wavelet transform is to represent the function or signal to be analyzed through a series of wavelet function expansion and translation combination. If multiple scale projection decomposition is performed in the time domain, analysis in various domains can be carried out [5, 6]. The advantage of wavelet analysis is that the size and shape of time window and frequency window can be changed by scalable translation, and finally the research purpose of local analysis in time and frequency domain can be achieved. The development of school education culture has changed the traditional teaching concept. The vision of modern teaching concept is not limited to the classroom but has taken a social perspective, changing the concept of “school is teaching”, emphasizing “open teaching,” “lifelong teaching,” “interactive teaching,” and “individualized teaching” [7]. The wavelet transform algorithm emphasizes the dialectical unity of teaching and learning, emphasizes the combination of the leading role of teachers in teaching and the main role of students in teaching, gives full play to the enthusiasm of both teachers and students, effectively utilizes all learning resources, teaching methods, and modern educational technologies, and stimulates students' internal drive and conducts effective learning. We can see that under the wavelet transform algorithm, school education culture has put forward higher requirements in terms of education scale and education quality.

Similar to the process of social modernization, the growth of instrumental rationality with the aid of scientific and technical forces furthers and deepens the process of school education and culture. This rational thought can be seen in the acceptance of the regularity of social development: the world as an orderly place that can be understood by human reason, and the belief, curiosity, and study of the general order and the natural laws that underlie it [8]. The wavelet transform algorithm consistently adheres to learning from teaching in the emotional education of cross-media narration and cultivates the students' emotions through experiencing the emotions of the lesson materials in the classroom. It promotes the students' sense of morality, justice, and beauty and gives them the opportunity to have greater emotional experiences, while also maximizing the instructional value of the reading course topics. The wavelet transform allows teachers to accurately communicate the cross-media narrative to students in the education culture teaching by ensuring that they properly comprehend the content in the textbook, the text's deeper meaning, and the author's thoughts and feelings [9]. The classroom environment should be harmonious, the effectiveness of teaching emotional identification, and the learning outcomes of the students should all be improved. At the same time, children should also sense the teacher's relationship with them and the teacher's kindness while learning.

The cross-media narration and emotional identification of school education culture under the wavelet transform is an education that fully exploits the potential of students, implements the education policy of all-round development, and focuses on cultivating talents who adapt to the market economy. In the teaching process, teachers who pass the wavelet transform infiltrate the basic knowledge of Chinese into the emotional cultivation of students, which is conducive to the emotional edification, personality development, and self-motivation of students. The main innovation points in the paper are the following: (1) this paper puts forward the implementation strategy of cross-media narrative and emotional education based on wavelet transform. After using wavelet transform to decompose the signals to be processed in cross-media narrative and emotion analysis, the interference noise is concentrated in the high-frequency wavelet coefficients, the corresponding amplitude is small, and the number of wavelet coefficients is large. But the useful part is opposite to the noise part. To sum up, it can eliminate the part with smaller wavelet coefficient of cross-media narration and emotional identity and retain the part with larger amplitude, so as to eliminate the noise interference correspondingly. At present, the threshold method can be applied to achieve this purpose. (2) This paper studies the meaning structure matrix of netizens' narrative text. Its core meaning is as a psychological process, which is different from the cognition of reflecting the objective things themselves. It reflects the relationship between the objective things and individual needs. By reflecting this relationship and through a series of attitude experiences, individuals form various personality characteristics, such as attitude, values, will, and quality. In the sense of psychology, emotion is a complex and unique psychological phenomenon unique to human beings.

## 2. Related Work

Taking emotional identity as the more fundamental cultural purpose of school education may have a more accurate connection with the theme of quality education put forward in our basic education. Quality can only be internal. Only when cognitive information is integrated into the emotional field and internalized into people's emotional personality can it be internalized into “human” things and become human quality. Emotion, with its living connection with individual life, its preexisting position over reason, and its advantage as human power system, opens the way to value reason.

Yu-xin et al., a preliminary investigation of the current situation of emotional education in school education culture will reveal that there are endless problems in emotional education. Of course, this is the result of the common restriction and influence of various factors such as society, culture, system, and social habits. At present, the phenomenon of students' high scores and low abilities, and the serious lack of emotional education, etc., has aroused widespread attention in the educational circles [10]. Tickoo argued that the educational environment in schools recognizes the rich artistic expression, emotional experience, and thought processes of its students. Try to grasp the rich social life and emotional realm of people by exploring the national psychology and the spirit of the times included in the works. All of these initiatives aim to represent the role that subjective emotion plays in reading instruction, promote the right value orientation, and help students connect with the text's vast range of human emotions [11]. According to Krishna et al., emotional identity is a crucial component of the entire educational process. Students can improve their ability to control their emotions, encourage them to have positive emotional experiences in their studies, life, and everything around them, form independent and sound personalities and personality characteristics, and truly become complete individuals with all-round development of moral character, intelligence, physique, and aesthetic feeling. This is done by respecting and cultivating students' social emotional qualities in the process of school education and culture [12]. Khare et al. through the analysis of basic theories such as philosophy, systematic science, brain science, psychology, emotional physiology, and pedagogy, the feasibility of emotional education in Chinese reading teaching is demonstrated, and the methods and ways of how to effectively implement and carry out emotional education in the actual school education and cultural teaching are explored [13]. Gupta et al. showed that emotional identity is fundamentally human life education and how a person can grow into a human being in a complete sense. Therefore, correcting the position of emotional identity in school education culture is required and must be realized by educational significance itself [14]. Goshvarpour and Abbasi think that the cultural concepts of school education, as opposed to emotional identity, are intellectual education and cognitive education. Only rational education refers to the education with the sole purpose of imparting systematic knowledge and developing rational ability, and with the help of rational means and tools such as language, concept, logic and science with fixed meanings [15]. Wang et al. nourish students' emotions with the rain of life, so that students can be educated from it. Sincerity, respect, and understanding are the elements of Tao Xingzhi's three qualities in treating students, and the key to the success of his school education and culture [16]. Choi and Kim think that emotion is a very complicated psychological phenomenon of human beings, so it has always been a weak field in psychology. Similarly, there are few researches on the theory and practice of emotion teaching. However, the research on emotional teaching strategies for school education culture is only scattered in related works or papers, which is not systematic enough [17]. Gramner and Wiggins in the content of school education and culture, clear, logical, and systematic scientific knowledge, theories, and professional expertise and skills are the main contents. In the organizational form of education, classroom teaching, and formal curriculum are the most basic and main organizational forms [18]. On the basis of emotional identity, AragO systematically expounds the psychological theory of using emotional factors to optimize teaching under the background of the interaction between cognitive and emotional information loops in school educational and cultural teaching activities. Advocating the teaching idea of promoting knowledge with emotion and enriching knowledge, so as to improve students' comprehensive, harmonious, and healthy development [19].

Based on wavelet transform, this paper studies the mechanism of cross-media narrative and emotional identity in school education culture. The cross-media narrative school education culture caters to the needs of different audiences for media selection and meets the requirements of audience's exploration, experience, and participation. Through cross-media, words, sounds, images, videos, and other means can be integrated to tell the charm of culture with vivid descriptions, vivid images, and delicate emotions, so that the audience can feel, know, and enter their minds and hearts. Through the practice of wavelet transform, it is proved that the subjective initiative of individual students is the fundamental power of their physical and mental development, and the ultimate goal of education is to stimulate students' learning potential. Teenagers' physical and mental development exhibits a variety of traits depending on their age under the culture of school instruction. Cross-media narrative emotional education in schools refers to instruction where teachers emphasize cognitive factors, and wavelet transform is used to elicit, mobilize, and satisfy students' positive emotional needs and cognitive needs through language, attitude, behavior, and other teaching variables to support the improvement of teaching objectives, the enhancement of teaching effect, and the optimization of the teaching process. Cross-media emotional and narrative instruction should be flexible enough to accommodate different phases of students' physical and mental growth as well as different disciplines with a variety of objectives and approaches. When teaching Chinese reading, we should pay attention to emotional education and develop efficient emotional education strategies to support the balanced and normal development of middle school students' emotions and personalities. This is in accordance with the characteristics and laws of middle school students' physical and mental development under the school education culture.

## 3. Method

### 3.1. The Concept and Characteristics of Cross-Media Emotion in School Education Culture

School education culture is not only a cognitive process but also a process of emotional will. Emotion is the core of nonintelligence factors. It not only regulates motivation, interest, will, and other factors but also promotes the development of intelligence factors. Therefore, in the overall development of human beings, emotion exists not only as a nonintellectual factor but also as an intermediary driving factor between cognitive factors and other nonintellectual factors. The impact of this tendency on education is undoubtedly negative: the backward spirit of scientific humanism leads to students having “rich” knowledge reserves, but their creativity and imagination are almost exhausted [20]. Students can get high scores as long as they bury themselves in hard work, but their study is not vivid and full of fun. In terms of academic tradition, there are three main dialogue contexts involved in the study of emotional expression phenomenon of new media events: first, in the field of communication, the media event theory and cultural analysis theory are used as the reference frame to analyze the transformation and reconstruction of the nature and social psychological structure of public events by new communication technology, as well as the mobilization mechanism of emotion in network events; second, in the field of sociology, it analyzes how emotion connects individual and collective, structure, and action in the network social movement and the network protest politics with the group events as the entry point; and the third is the rediscovery of the value and role of emotion in the revolutionary movement in the field of history [21].

In cross-media events, emotional expression based on personal cognitive paradigm and social “moral grammar” permeates the actor's own life experience and social experience. In the meaning structure model of Figure 1, the narrator puts Yang Jia's attack on the police into a common narrative structure in traditional Chinese society where individual's dignity is humiliated by unscrupulous officials and the power system behind it, so that there is no way to rise up and resist, thus endowing Yang Jia's attack on the police with moral legitimacy and cultural identity. In the face of power oppression, Yang Jia's tragic “heroic” resistance and the mutual penetration of netizens' own experiences and encounters in the world of life stimulated the surging blood and surging emotions of netizens. In the praise of Yang Jia, netizens vented their resentment, completed “imagined revenge”, and regained their affirmation and recognition of themselves. The traditional morality and culture in the meaning matrix are cited by netizens as a project in value, providing meaning explanation, and value confirmation for the police attack and their own emotional expression. The meaning structure matrix of netizens' narrative text is shown in Figure 1.

Its core meaning is as a psychological process, which is different from the cognition that reflects objective things themselves, and it reflects the relationship between objective things and individual needs. By reflecting this relationship and through a series of attitude experiences, individuals form various personality characteristics, such as attitude, values, will, and quality. From the psychological point of view, emotion is a complex and unique psychological phenomenon peculiar to human beings.

Cross-media narrative of school culture and emotional analysis with emotional analysis coefficients such as

(1) $$\begin{array}{c} S_{2}=\sum \left[h_{k}S_{2}\right],\\ W_{2}f=\sum \left[g_{k}S_{2}\right], \end{array}$$

where *S*_2_ is a smooth operator; *h*_*k*_ is the signal to be analyzed. *W*_2_*f* is the emotional transformation of signal *f*; *g*_*k*_ and *S*_2_ are coefficients of *H*(*w*) and *G*(*w*), respectively.

The quadratic spline scaling function is adopted, which is the first derivative of the smoothing function. The emotion coefficient is shown in

(2) $$\begin{array}{c} H\left(z\right)=\frac{\left(1+3^{-1}\right)}{4},\\ G\left(z\right)=\frac{\left(-1-3z^{-1}\right)}{4}. \end{array}$$

The final coefficients are *h*_0_ = 1/4, *h*_1_ = 3/4, and *h*_2_ = 3/4.

The relationship between the mixed signal and the source signal can be described by the formula

(3) $$\begin{array}{c} x\left(k\right)=\text{As}\left(k\right). \end{array}$$

In addition, when the source signal *s*(*k*) and the mixing matrix *A* are unknown, the solution mixing matrix *w* is obtained by observing the data vector **x**(**k**), and the transformed output is as follows

(4) $$\begin{array}{c} y\left(k\right)=W\cdot x\left(k\right) \end{array}$$

where *y*(*k*) is the estimation of the source signal *s*(*k*) and *w* is the inverse matrix of the mixing matrix *A*.

To treat emotional education with a modern comprehensive way of thinking, it has the basic characteristics different from logical and rational education, which are mainly scientific, adaptive, creative, and interesting.

1. Adaptability

The traditional education mode is the preset goal, the introduction goal, and the expectation goal. This kind of teaching mode separates the educational goal, the content, and the educated individual, and makes it difficult to find the connection point between them in the actual operation process.

(2) Scientific nature

The scientific nature of emotional education is the common feature of all aspects and links of emotional education. Contemporary emotional education is based on the recognition of the historical inevitability and rationality of the development of modern science. Therefore, it does not avoid scientific rational education.

(3) Interest

The characteristics of interest in emotional education are as follows: in the process of emotional education, starting from the emotional aspects of students, students' internal learning interest is aroused, and students' interest quality is developed in the learning process. Students' interests and emotions always restrict and promote each other and exist together. Emotional education must grasp the internal interest of students' learning and create it as a basic condition.

In view of the cross-media emotional and psychological development characteristics of school education culture, the emotional functions of various constituent elements of the teaching process are integrated to give full play to the role of emotional power, mediation, organization, and so on, and stimulate students' positive emotions, so as to achieve the educational model of making students' feelings and knowledge progress together, forming a healthy personality and all-round development.

### 3.2. Implementation Strategy of Cross-Media Narration and Emotional Education under Wavelet Transform

The two basic properties of wavelet are, firstly, the existence of compact support or approximate compact support in time domain. Secondly, the positive and negative changes alternately, so that the DC component is zero. The information content of signal continuous wavelet transform coefficients is redundant, which makes the algorithm more difficult. Therefore, in order to reduce the calculation amount under the principle of no distortion, continuous wavelet transform can be discretized in practical application. In particular, it is only the discretization of scale factor and time shift factor, but not the time variable. Among all noises, the influence is the most significant. Therefore, baseline drift should be eliminated first. As for the interference and burying of power frequency and EMG signals in ECG, the signal waveform changes, and even the characteristic wave cannot be detected, which ultimately affects the emotion recognition result. Therefore, these noises must be avoided. In this paper, wavelet transform is used to remove the above noises. The teaching strategy of school education culture is to grasp the regularity of cross-media narration and emotional identity of school education, which is reflected by teaching methods, teaching modes, and teaching means. To successfully complete teaching tasks and achieve teaching objectives, Chinese teaching cannot be separated from the proper use of teaching strategies. Emotion education focuses on people's development and attaches importance to the role of emotion in Chinese teaching. Therefore, the use and arrangement of teaching strategies should also focus on students' life activities, focusing on the embodiment of culture and emotional development. Although the traditional teaching theory has pointed out the role of emotion, it regards emotion as an auxiliary means of cognition, not as a psychological ability parallel to cognitive ability, and it has not been included in the teaching category and studied. It is an urgent task for us to promote the development of media convergence and build the whole media. We should fully grasp the trend and law of media convergence, adhere to the direction of integrated development, speed up the transition from addition stage to integration stage, and create a number of new mainstream media with strong influence and competitiveness. It is necessary to promote the in-depth development of media integration, speed up the construction of an integrated all-media communication pattern, and significantly improve the quality and level of positive publicity through innovations in ideas, contents, forms, methods, and means.

Therefore, after the signal to be processed is decomposed by wavelet transform, the interference noise is concentrated in the high-frequency wavelet coefficients, and its corresponding amplitude is small, and the number of wavelet coefficients is large. However, the useful part is contrary to the wavelet coefficients of the noise part. To sum up, the part with small wavelet coefficients can be eliminated, and the part with large amplitude can be kept, so that noise interference can be eliminated correspondingly. At present, threshold method can be used to achieve this goal. According to the infiltrating function of the teaching situation of cross-media narration and emotional recognition of school education, in Chinese teaching, teachers should start from the needs of teaching, create specific scenes or atmosphere suitable for teaching content, and bring students into the society and nature described in the works, so that students can get emotional experience and aesthetic edification in a subtle way, and change “this situation and this situation” into “my love and my scene” in Chinese teaching. The experiment and research of modern emotional psychology have proved that cross-media narrative school education emotion has a broad and profound biological basis in forming people's subjective psychology. At the same time, when defining the concept of emotion, we pay attention to the sociological basis of emotion through wavelet transform. Because human beings are social beings, they have powerful rational cognitive function, rich meaning generation ability, and value selection and identification mechanism. Besides the mainstream media, national diplomacy, government publicity, enterprise marketing, nongovernmental organization communication, and individual communication are the ways to spread excellent traditional culture, followed by the diversification of narrative content. Besides the feature films of the dominant content of Chinese excellent traditional culture, other diversified contents such as traditional medicine, folk crafts, cultural education, painting art, food, and costume design should also be developed. The following is the implementation strategy of cross-media narrative and emotional education, as shown in Figure 2.

Teachers must put in a lot of effort to moderate their use of language in the classroom by fusing cross-media narration with appeal and persuasion in the classroom. However, when characterizing the instructional environment, the terminology used should take into account a number of factors. The language should be vibrant first. In addition to being precise and consistent, the instructional language should also be engaging. Teachers should therefore use vivid language to describe or explain in accordance with the content of cross-media narrative and school education culture teaching materials, combined with reality, when instructing using wavelet transform.

Let the cross-media narrative be *ψt* ∈ *L*(*R*), that is, the square integrable function. If it meets the following admissibility conditions, it is shown in the formula.

(5) $$\begin{array}{c} C_{\psi }=\int \frac{\left|\psi \left(\omega \right)\right|}{\omega }, \end{array}$$

where *ψt* is a basic cross-media narrative emotion analysis.

After the expansion and translation of the school education culture *ψt*, the formula is obtained

(6) $$\begin{array}{c} \psi_{\alpha }t=\alpha ,\tau \in R,\alpha >0, \end{array}$$

where *α* > 0, translation factor *τ* are nondiscrete values, and *ψ*_*α*_*t* are continuous emotional values.

Let *f*(*x*) also be square integrable, be *f*(*x*) ∈ *L*(*R*), and extend *f*(*x*) under *L*(*R*) under the above emotional values. As shown in the formula, it is the continuous wavelet transform of *f*(*x*).

(7) $$\begin{array}{c} \text{WT}\left(\alpha ,\tau \right)=\left\{f\left(t\right),\psi_{\alpha ,\tau }\right\}dt, \end{array}$$

where *ψ*^∗^(*t*) is the complex conjugate of *ψ*(*t*).

If the emotional education of *f*(*x*) is transformed into WT(*α*, *τ*), the *f*(kx) is transformed into the formula.

(8) $$\begin{array}{c} \frac{1}{\sqrt{k}}{\text{WT}}_{f},c>0. \end{array}$$

Transform the numerical value of emotional education into a formula

(9) $$\begin{array}{c} {\text{WT}}_{f}=\frac{1}{\sqrt{\alpha }}f^{*}\bar{\psi }. \end{array}$$

Type, $\left(1/\sqrt{\alpha }\right)f^{*}\bar{\psi }$. Therefore, emotional education transformation can be regarded as the convolution calculation of emotional analysis and school education culture.

There is a subtle relationship between emotions and people's cognition, because “in the process of understanding things, people will inevitably experience different emotions because the neural processes caused by things of different nature in their own brain hemispheres and other neural processes that have occurred and the related dynamic stereotypes have different interactions. These emotional factors, in the process of cross-media narration and school education and teaching, have a comprehensive impact. In the teaching of wavelet transform, the role of emotional factors should be mobilized and utilized. Using wavelet transform can help to cultivate students' good psychological and emotional quality, improve students' interest in learning, and increase their understanding of the content taught, so as to achieve the purpose of improving the teaching effect. It is often said that “I am old, I am old, I am young, and I am young” is actually an emotional understanding that people seek.

## 4. Result Analysis and Discussion

This paper analyzes the cross-media narrative and emotional analysis of school education culture and studies the heart rate. The heart rate variability signal was obtained by emotion analysis interval spectrum. It can be seen from the above that the obtained heart rate variability signals are nonuniformly spaced. After cubic spline interpolation, emotion signals with uniform intervals are obtained, and then resampled. Finally, the uniformly spaced emotion signal after resampling is obtained. The resampling frequency is 5 Hz and the interval is 0.28 s, as shown in Figure 3.

In this paper, the cross-media narrative and emotional identification of school education and culture are used for the experiment. Firstly, the R wave is accurately located by the characteristic wave detection method mentioned above, and then the corresponding RR interval is obtained by subtracting the abscissa of the peak value of R wave, which is an unequal interval emotional characteristic signal, as shown in Figure 4.

In this paper, the emotional identity analysis samples are directly operated under the school education culture, so it is not limited by specific problems and has strong generalization ability. In addition to strong global optimization ability, it is not affected by function derivation and continuity, and the search direction can be adjusted according to the search situation. The experimental results are shown in Figure 5.

As shown in Figure 5, the group with the best fitness curve in the process of multiple optimization of parameter C and parameter value, in which the termination number is 54, the population number is 26, the cross validation accuracy rate is 94.5543%, and the optimal parameter C and parameter value are 1.8631 and 2.273, respectively.

This paper compares and analyzes the ECG time domain features, ECG wavelet features, conventional heart rate variability time-frequency features, and heart rate variability features extracted by wavelet-ICA algorithm. The results are shown in Table 1.

As can be seen from Table 1, the recognition results of emotional feature sets of various school education cultures all reach over 90%. Among them, for the recognition of happy, angry, and fearful emotions, wavelet-ICA algorithm HRV feature recognition achieves the highest recognition rate, reaching 92.4%, 93.74%, and 95%, respectively; For sad emotion recognition, ECG time domain plus wavelet feature recognition ability is the strongest, which is 95%. Moreover, in the table, the highest recognition rate is the recognition of angry emotion by HRV features of wavelet-ICA algorithm.

When studying and analyzing the emotional characteristics of school education and culture, each kind of emotional recognition is performed 55 times, among which the classification accuracy rate is 55 times, and the ratio of training set to test set is 4 : 1. Each sample is randomly selected, and the corresponding sample labels correspond one to one. When a single emotion is classified, the emotion to be identified is marked as 1, and the other emotions are of the same kind and marked as 2. In this paper, the emotions of happiness, anger, sadness, and fear are identified, respectively. The simulation results of emotion recognition are shown in Figure 6, and the recognition accuracy rate is 96%.

This experiment selects and optimizes the emotional features of school education and culture through literature [5], literature [9], and this method. The following analysis is made on the recognition results of each feature selection algorithm and emotional feature set. For emotional recognition of happiness and fear, the feature rate of this method reaches the highest recognition rate, which is 95.6% and 94.5%, respectively; For the recognition of anger, ECG time domain + wavelet feature has the strongest recognition ability, 94.75%; among them, the highest recognition rate is the recognition of sad emotion by wavelet features. As shown in Table 2.

In this paper, the sampling rate of emotional ECG signal is 1000 Hz, and the emotional ECG signal is decomposed by 7-layer wavelet. The scale selection is based on the frequency component of the ECG signal and the signal sampling rate. It is known that the sampling frequency of the ECG signal collected in this paper is 1000 Hz. The frequency information corresponding to each level after wavelet decomposition is shown in Table 3.

As can be seen from Table 3, the frequency band of ECG signal is 0.07~110 Hz, among which the QRS complex characteristic analysis shows that it is mainly concentrated in 5~45 Hz, while the center frequency is concentrated in 21 Hz. At the same time, in order to eliminate high-frequency interference and low-frequency baseline drift, this paper selects D4~D5 wavelet information for statistical calculation, and calculates the mean, median, variance, minimum, maximum, the difference between minimum and maximum, and the above values of first-order difference, and obtains 36 wavelet time-frequency characteristics. In this experiment, the emotional features of school education culture were selected and optimized by the methods in literature [5], literature [9], and this paper. For the error rate obtained by the identification results of each feature selection algorithm and emotional feature set, the error rate changes of the three methods were obtained as shown in Figure 7.

In this experiment, the error rate of emotional feature recognition is tested through literature [5], literature [9], and this method. As can be seen from Figure 7, the recognition results of each feature selection algorithm and emotional feature set are analyzed as follows. Among the three methods, the error rate of this paper is the lowest, with the highest error rate of 46.8%, followed by the method of literature [5], with the highest error rate of 64.8%, and finally the method of literature [9], the highest error rate is 71.8%. It can be seen that this method is the most suitable to identify the emotional characteristics of school education culture.

## 5. Conclusions

Because of the predominance of cognitive education in the past, individuals either overlooked the cross-media narrative of school culture and the emotional education of emotional identity or integrated it into the overall education. Both the culture of school instruction and the overall development of individuals are unavoidable prerequisites. The emphasis on understanding education via the emotional and cross-media narrative features of school culture is meant to address the imbalance in teaching, not to discount or deny the cognitive aspects of instruction. The wavelet transform algorithm is primarily used in this paper to study the cross-media narrative and emotional identity of school education culture. The study reveals that, of the three ways, this one has the lowest mistake rate, with the maximum error rate being 46.8%. The other two methods are the method of literature [5], which has the highest error rate of 64.8%, and the method of literature [9], which has the highest error rate of 71.8%. It is clear that this approach works best for determining the emotional traits of school culture. We cannot cultivate the critical role of healthy and perfect emotion in the physical and mental development of teenagers and put it into practice in teaching work, unless we fully utilize the wavelet transform algorithm to pay attention to the importance of cross-media narration and emotional identity of school education culture. Only then will our education be able to cultivate a generation of genuinely high-quality talents, and our society will be able to move steadily toward civilization.

## Figures and Tables

**Figure 1:** Meaning structure matrix of netizens' narrative text.

**Figure 2:** Implementation strategies of cross-media narrative and emotional education.

**Figure 3:** Uniform emotional signal after resampling.

**Figure 4:** Unequal interval emotional characteristic signals.

**Figure 5:** The process of emotional identification optimization in school education culture.

**Figure 6:** Accuracy of emotion recognition.

**Figure 7:** Error rate of emotion recognition.

**Table 1:** Analysis of classification results of emotional feature set.

Features	Happy	Anger	Sadness	Fear
Time domain	92.4	93.4	92.4	93.5
Wavelet	93.4	94.4	93.4	93.24
Time frequency	93.4	92.74	94	93.5
Time domain + wavelet	92.4	93.74	94.5	95

**Table 2:** Analysis of emotion recognition results.

Features	Literature [5]		Literature [9]		Method in this paper	
	Happy	Fear	Happy	Fear	Happy	Fear
Time domain	92.4	93.5	92.5	94.2	93.1	95.2
Wavelet	91.4	92.24	92.25	93.6	92.56	93.1
Time frequency	92.5	93.2	94	94.2	94.6	94.5
Time domain + wavelet	93.4	94	93.6	95	94.2	95.6

**Table 3:** Frequency band range of ECG signal components.

Decomposed component	Band range
D1	252~502
D2	126~252
D3	64.3~126
D4	32.26~64.4
D5	16.12~32.24

## Data Availability

The data used to support the findings of this study are available from the corresponding author upon request.
